The article "From darkness to light: Unveiling the asymmetric nexus between energy poverty and environmental quality in South Asia" was retracted in 2025. Reasons: unreliable results or conclusions; concerns about the peer review; concerns about the authorship.

# From darkness to light: Unveiling the asymmetric nexus between energy poverty and environmental quality in South Asia

**DOI:** 10.1016/j.heliyon.2024.e27100

**Published:** 2024-02-24

**Authors:** Jifa Rao, Sajid Ali, Raima Nazar, Muhammad Khalid Anser

**Affiliations:** a School of Architecture and Art, Central South University, Changsha, China; b School of Economics, Bahauddin Zakariya University, Multan, Pakistan; c Department of Economics, The Women University Multan, Pakistan; d School of Business, Xi'an International University, Xi'an, 710077, Shaanxi, China

**Keywords:** Energy poverty, Quantile-on-quantile estimation, Environmental quality

## Abstract

Energy poverty alleviation has emerged as a critical economic problem in recent years. Given the enormous number of people without essential energy services, a crucial concern is whether providing universal access to electrification will considerably affect environmental quality. The present research evaluates the asymmetric energy poverty-environmental quality nexus in South Asian economies. Previous works adopted panel data techniques, resulting in distinctive conclusions about the energy poverty-environmental quality nexus, irrespective of the truth that several nations could not establish such a correlation separately. This research, conversely, applies the Quantile-on-Quantile methodology, which enables independent determinations of time-series interconnection in all nations to offer worldwide yet economy-particular evidence concerning the relationship between the variables. The results indicate that energy poverty degrades environmental quality in most selected economies at particular data distribution quantiles. Moreover, the findings disclose that the ranks of asymmetries between the variables change by country, emphasizing the requirement of governments to take special care when accepting policies linked to energy poverty and environmental quality.

## 1 Introduction

Poverty alleviation is a primary goal of the sustainable development goals (SDGs), aimed at fostering long-term socio-economic development, as highlighted by Zhao, Jiang, Dong, & Dong [1]. Within this framework, energy poverty (*EP*) emerges as a critical issue in the energy sector, often seen as a distinct facet of poverty, is the inability to access sufficient energy to face bare necessities [2]. The concept of *EP* is dynamic and varies based on its measurement criteria, leading to numerous interpretations and definitions, indicating an ongoing debate over its precise conceptualization. The term *EP* was initially used in the early 1970s during a fuel usage campaign in the UK, focusing on the lack of ability of households to yield essential energy services. Expanding on this, Boardman [3] determined *EP* to be households' incapacity to afford essential energy services. This definition was further refined by Hills [4], who described *EP* as a “low income-high cost,” emphasizing the financial strain households face in accessing energy. Additionally, Churchill & Smyth [5] broadened the scope of *EP*, associating it with households' failure to sustain associations to essential energy-related facilities or to sustain adequate home heating. This evolving understanding of *EP* reflects the issue's complexity, encompassing various economic, social, and environmental dimensions.

The multifaceted nature of *EP* underscores its significance in the broader context of sustainable development, as it intersects with several other SDGs, including those related to health, education, and environmental sustainability [6]. Addressing *EP* is crucial for achieving holistic socio-economic development and ensuring equitable access to energy resources across different socio-economic groups. However, the definitions of *EP* discussed above are essentially linked to energy costs and hence apply mostly to developed economies. The International Energy Agency established a much more appropriate notion for underdeveloped economies, which defines *EP* as a scarcity of neat fuel, electricity, and energy services, and a high reliance on conventional fuels [7]. Given the harmful effects of *EP* on economic well-being, most countries throughout the world have made significant efforts to reduce *EP* during the last few decades, with notable results. The global population without availability of electricity has continuously decreased from 1685 million in 2000 to 775 million in 2019 [7,8].

Many economists are concerned about the environmental consequences of *EP*, notably the implications of carbon dioxide emissions (*CO*_*2*_). People's inability to get clean fuels, their reliance on conventional energy sources (e.g., firewood and biomass), and insufficient cooking devices all contribute to environmental degradation [9]. Nations with increased energy usage significantly influence growth, human development, and pollution [10,11]. People who suffer from *EP* have insufficient energy to live a comfortable and healthy life. Thus, they will inevitably require more energy to escape such a horrible predicament. However, increased energy consumption degrades environmental quality (*EQ*) unless the extra energy usage is supplied by non-carbon energy (e.g., renewable energy) or wholly compensated by decarbonization by the non-energy poor people ([12]; Haldar et al. [13]. People in *EP*, in general, might not manage to acquire carbon-free energy sources like solar panels on their own [14,15]; thus, *EP* reduction initiatives are more likely to increase *CO*_*2*_ if appropriate countermeasures are not implemented [16,17].

Exploring the *EP-EQ* link is quite difficult. Is it true that in South Asian economies, *EP* degrades *EQ*? Does a non-linear bond exist between *EP* and *EQ*? How do *EP* and *EQ* patterns diverge between economies as data distribution points change? What are the policy repercussions of environmental changes originating from *EP*? An investigation of the studies suggests that these are ignored issues, and to the extent of our awareness, limited works that tackle the abovementioned problems are accessible. The extension of ongoing research to recent literature might be categorized into three types: First, many empirical works on the linkage between *EP* and *EQ* have been done in the past (for example, [1,16,18,19]). To our awareness, no past work has investigated the association of the variables above in South Asian countries.^1^ Second, past studies concentrated on panel data methodologies to identify the *EP-EQ* link, disregarding the truth that other economies possess no indication of this type of linkage autonomously [[20], [21], [22]]. Conversely, this research employs the QQ method to bring global yet economy-related facts on the bond between *EP* and *EQ*. The QQ model evaluates each economy's time-series dependency distinctly. The *EP-EQ* nexus possesses many features that make it challenging to study applying old techniques (for example, quantile regression and OLS). Customary parametrical estimations resist alterations and might have not consider for heterogeneity of slopes [23]. Consequently, assessing the effect of *EP* on *EQ* necessitates the implementation of a strong, innovative econometric instrument, like QQ, that can easily tackle the above-mentioned issues [24].

Past research also assessed single parameters with positive or inverse signs across their respective complete sample data distribution [21,22,25,26]. On the contrary, this research defines that sole indicators (positive or negative) can be derived along various data quantiles. When the economy is in decline, the influence of *EP* might be varied from when it is thriving. Equally, the impact of higher *EP* ranks over *EQ* could diverge from that of lower *EP* ranks. As *EP* capability uplifts, the bond between *EP* and *EQ* may become more dynamic and complicated. Because dispersion features induce non-linear or asymmetric trends in economic variables, we hypothesize an asymmetric *EP-EQ* nexus [23,27]. We can also find co-movements (causalities) of *EP* and *EQ* at various data quantiles (i.e., mid, topmost, or bottom). While *EP-EQ* link changes, our research's single-country technique might give critical economy-particular proposals for attaining economic, social, and political considerations at the lowest, median, and high grades of *EP* and *EQ* quantiles.

The choice of South Asian economies as the focal point of our research is founded on their unique developmental, economic, and environmental characteristics. This region, comprising rapidly underdeveloped economies containing Pakistan, Nepal, Sri Lanka, India, and Bangladesh, presents a distinctive scenario of *EP* amid rapid economic growth, as Amin et al. [28] noted. These countries are transitioning from agrarian to more industrialized economies, a shift that significantly affects the energy consumption patterns and *CO*_*2*_, offering a crucial perspective for understanding the effect of economic development on environmental sustainability, as explored by Katekar, Asif, & Deshmukh [29]. The interplay of their similar political, economic, and social systems provides a rich comparative backdrop. Our methodological choice, particularly the Quantile-Quantile (QQ) estimation, as suggested by Yu et al. [23], effectively addresses the heterogeneity and cross-sectional dependence unique to these economies. This approach allows for a detailed, country-specific analysis, crucial for accurately capturing the nuances of the association between energy usage, economic growth, and environmental impact in South Asia. Economic integration through economic, social, and political development is a critical component of various economies. Contemporary history has shown that volatility shocks in one economy could quickly spread to other nearby nations [30]. Additionally, the energy sector depends on its neighbors' energy sectors and external and internal shocks [31]. Hence, the first point in our work is to investigate each nation distinctly to evade the abovementioned difficulties. Fourth, regardless of their profound interconnectedness, these nations can occasionally stay very independent, as each has its energy consumption patterns [28]. Consequently, QQ, an econometric tool, is needed for the empirical modeling approach to consider heterogeneity among economies. Hence, the research's findings can give an exhaustive picture of the bond between the preceding variables that may be tough to get by employing traditional econometric methodologies. This study will also support policymakers and governments in developing plans at different *EP* and *EQ* ranks. Ultimately, this investigation will lead the pathway for future research on this topic and its ramifications for other groups of nations.

The remaining portion of the present research is arranged as follows: Section 2 gives the review of previous empirical studies while Section 3 depicts the theoretical framework and hypothesis of the study. Section 4 defines the data, whereas Section 5 introduces the research technique. Section 6 gives the initial and main findings with a detailed discussion. In the end, section 7 concluded the study with some future implications.

## 2 Literature review

*EP* has gained a great deal of consideration in current years as environmental concerns have risen. With the increased focus on *EP* in recent years, many economists have looked at the association between *EP* and pollution [19,20,22,32,33]. In the presence of elevated *EP*, Haldar et al. [13] examined EP in Sub-Saharan Africa, using system GMM and 3SLS models to explore the impact of governance and renewable energy. It found that government expenditure reduced EP and highlighted the importance of strong institutions and renewable energy integration in addressing regional energy challenges. Reyes et al. [16] proposed that extensive wood consumption for cooking and heating worsened air quality in Chile. Moreover, González-Eguino [34] indicated that using organic matter or animal dunk in inefficient cookstoves resulted in enormous indoor pollution. Barron & Torero [32] explored the association between household electrification and indoor air pollution in El Salvador. It was concluded that household electrification lowered indoor air pollution due to low paraffin consumption. Without electricity, most houses relied on paraffin for lighting, resulting in dangerous amounts of soot emissions for those exposed. PM 2.5 concentrations were 63% lower in residences compelled to connect to the electricity grid than in those not. Similarly, Crentsil et al. [35] also claimed that *EP* in underdeveloped economies negatively affected *EQ*. In the context of the *EP-CO*_*2*_ association, Sovacool [36] documented that *EP* contributed to household pollution, the environmental consequences of *EP* encompassed GHG emissions. In another study, Pereira et al. [9] observed that switching to clean energies (i.e., reducing *EP*) minimized *CO*_*2*_. Furthermore, Chakravarty & Tavoni [37] evaluated the relationship between *EP* and *CO*_*2*_, inferring that *EP* was inextricably linked to *CO*_*2*_ reduction and that neither the goal of eliminating *EP* nor carbon reduction could be accomplished independently, which was supported by the empirical work of Ürge-Vorsatz & Herrero [38].

Ehsanullah et al. [20] estimated the energy insecurity-*EP*-climate change nexus in G 7 economies. Data Envelopment Analysis (DEA) results showed that Canada had the highest EP index score, indicating that Canada has a stronger capacity to deal with economic development, energy self-sufficiency, and environmental performance than other G7 economies. France and Italy came in second and third place, respectively. Japan scored in second place with 0.50 EP index points. Hassan et al. [19] investigated the *EP-CO*_*2*_ nexus in BRICS economies. Continuously updated biased correction and continuously updated fully modified techniques were used by selecting panel data from 1980 to 2016. It was found that *EP* increased *CO*_*2*_ levels in these economies. Zhao et al. [1] explored the dynamic effects of *EP* on *CO*_*2*_ in 30 provinces of China with the aid of the generalized method of moments (GMM) technique. Although there were substantial disparities in *EP* among various locations in China, the country's *EP* level declined from 2002 to 2017. Moreover, *EP* accelerated the growth of *CO*_*2*_. Similarly, Okushima [18] measured the basic carbon needs of people in Japan and found that people suffering from *EP* required more carbon emissions than affluent populations to fulfil their basic energy needs. In another study, Zhao et al. [33] analyzed the *EP*-green growth nexus by employing the panel data of 30 Chinese provinces. It was found that *EP* eradication and increasing technological innovations effectively promoted green growth. In the same way, Bilgili et al. [22] scrutinized the energy access-*CO*_*2*_ damage nexus by using data from 36 Asian countries from 1997 to 2017. The panel quantile regression findings revealed an inverse link between energy access and *CO*_*2*_ damage.

### 2.1 Research gap

As per the literature above, previous studies concentrated on the overall effect of *EP* on the environment and have not study the relationship between distinct quantiles of the variables. Moreover, these inquiries have uncovered a symmetric connection between these variables. Nevertheless, the exclusion of potential nonlinear influences might neglect crucial nuances, potentially resulting in a misinterpretation of the outcomes. In previous research, panel data has frequently been favored over time-series data despite encountering challenges containing generalization difficulties, computation problems, and inadequate selection of the model. The heterogeneity in *EP* in panel data makes it unfeasible to calculate the average effect of *EP*-induced *EQ* for entire economies. The current study contributes to fill this research gap by employing the Quantile-on-Quantile methodology, allowing for distinct examinations for each economy individually. This approach can enhance our comprehensive understanding of the asymmetric relationship between various quantiles of both *EP* and *CO*_*2*_.

## 3 Theoretical framework and hypotheses

Though *EP* cannot be totally separated from conventional poverty reduction, its independent evaluation is vital for a variety of reasons. When household incomes rise, they tend to invest in new technologies, high-quality fuels, and renewable energy. This transition is referred to as the energy ladder. Moving up the ladder is related to reduced poverty, health difficulties, and pollution, as well as improved energy efficiency, gender equality, and education level [35]. Access to clean fuels and power does not always entail a move to clean alternatives, as many homes simply cannot afford it. A lack of alternatives may result in low-quality energy usage at greater costs [22]. Various theories and empirical findings explore the multifaceted nature of energy access and its environmental implications. Central to our discussion is the concept of *EP*, which encompasses not just the lack of access to advanced energy services but also its broader impact on living conditions and economic development [39]. This concept is pivotal in understanding the unique energy dynamics in South Asia. The Energy Ladder theory provides a foundational perspective as expounded by Van der Kroon, Brouwer, & Van Beukering [40]. It suggests a progression in energy usage patterns with increasing income, where households move from relying on traditional biomass to modern fuels. This transition is critical in understanding EP reduction in South Asia but is often characterized by asymmetries. These asymmetries arise from the region's diverse socioeconomic and geographic landscapes, as Sovacool [36] claims, where factors like income disparities, urban-rural divides, and varying energy policies influence energy access and consumption patterns differently across and within countries.

Trade-off theory argues that a trade-off exists between attempts at poverty elimination and *EQ* improvement. The exploitation of natural resources and *EQ* are emphasized as essential driving forces in the struggle against poverty. The main factors of *EP* are production expansion, low household incomes, high energy prices, poor residential energy efficiency, industrialization, and urbanization. The primary input of all of these crucial factors is energy demand. Around 80% of the global energy needs are fulfilled by fossil fuels, including oil, coal, and natural gas [38]. The utilization of fossil resources is the primary source of GHG emissions (particularly *CO*_*2*_), which cause climate change and global warming. This framework creates a conflict between global warming mitigation and poverty alleviation strategies. In general, it is believed that it can be accomplished by minimizing the demand for fossil energy and encouraging renewable energy (Sarkodie & Owusu, 2021). Combating *EP* is inextricably tied to the type of economic development and society we desire. This is a choice between an economy that aims to eliminate inequality, and promote sustainable development and social justice or stressing only market-led growth without thinking of winners and losers [36]. Many developing countries are still stuck in policies that support some energy sources. These subsidies are not largely made up of direct or pre-tax energy subsidies. They usually consist of inefficient amounts of energy taxation. These can have detrimental social and environmental consequences, such as local air pollution and associated health concerns, increased GHG emissions, clean energy sources, low investments in energy efficiency, and countries' continued reliance on imported energy sources [41].

The association between poverty and *EQ* can also be analyzed through the lens of ‘win-win’ and ‘trade-off’ hypotheses. The win-win theory claims that poverty alleviation and *EQ* enhancement occur concurrently. The win-win hypothesis is also maintained by the environmental Kuznets curve (EKC) hypothesis introduced by Grossman & Krueger [42]. The scale effect of EKC hypothesis causes pollution to rise in the early phase of economic growth [43]. This hypothesis is relevant in exploring how economic growth linked to energy access impacts *EQ*. However, the continuing process of economic growth and increase in income also influence the economy's structure and technology. When structural and technical effects develop, the ecosystem and natural assets are utilized more effectively, innovations and clean technologies emerge, and public awareness of climate issues grows [44]. Poverty diminishes during this growth process, which leads to a decrease in *CO*_*2*_ [45,46]. However, the direct application of the EKC hypothesis to South Asian contexts requires careful consideration. Studies like Arouri et al. [47] indicate that the linkage between energy consumption, economic growth, and environmental impact may sometimes follow a different EKC pattern in developing regions, suggesting a need for a nuanced application of this hypothesis in South Asia. Therefore, our theoretical framework aims to dissect the intricate and often asymmetric relationships between reducing *EP* and improving *EQ* in South Asia. It considers the unique challenges and dynamics of the region, such as the varying stages of economic development, diverse energy resources and policies, and environmental priorities. By integrating these theoretical insights and empirical findings, the framework provides a wider apprehension of how *EP* reduction strategies might be aligned with environmental sustainability goals in the South Asian context. Based on the theoretical and empirical evidences of *EP-EQ* nexus, the following hypotheses can be formulated.

H1 *EP* has a significant and negative impact on *EQ*.

H2 *EP* has an asymmetric effect on *EQ*

H3 The impact of *EP* on *EQ* changes across various quantiles of the data distribution.

## 4 Data

This study evaluates the *EP-EQ* nexus for South Asian countries.^2^ The dataset utilized in our investigation has two variables. *CO*_*2*_ is an independent variable used as a proxy for *EQ* since it significantly raises air pollution [1,19]. Energy poverty (*EP*) is used as an independent variable. Over the years, numerous economists have tried to measure *EP* through various methods (as already discussed at the start of the study); however, no consensus has been reached yet. Therefore, we measured *EP* by taking the people without access to electricity (% of the population), followed by the research of Amin et al. [28]. The data for *EP* and carbon emissions is attained through the World Bank (https://databank.worldbank.org/) for 1996–2019. Table 2 shows the description of variables and data sources. The list of signs and acronyms employed in ongoing work is listed in Table 1 at the very beginning of the research.

**Table 1:** The list of acronyms and symbols.

Acronym or Symbol	Narration	Symbol or Acronym	Narration
EP	Energy poverty	OLS	Ordinary Least Squares
EQ	Environmental quality	ADF	Augmented Dickey-Fuller
QQ	Quantile-on-Quantile Estimation	μ_t_^ɸ^	Quantile error term
QR	Quantile regression	h	Bandwidth parameter
J-B	Jarque-Bera	τ	τ^th^ quantile of energy poverty
CO_2_	Carbon dioxide emissions	$\rho_{\varphi }$	quantile loss function
Sup_τ_ |V_n_(τ)|	Supremum norm values of coefficients (α and γ)	SDGs	Sustainable development goals

**Table 2:** Variable description and data sources.

Variable	Symbols	Measurement	Data Sources
Energy poverty	EP	People without access to electricity (%)	World Development Indicators
Carbon dioxide emission	CO_2_	kiloton (kt)	World Development Indicators
Environmental quality	EQ	Represented by the amount of *CO*_*2*_ emissions (Low levels of emissions show improved environmental quality and vice versa)	World Development Indicators

## 5 Econometric technique

In the current study, the evaluation of the econometric tool used is negotiated in the ongoing section, where a quantile cointegration test is exerted to consider the long-run bond between the variables. Additionally, the estimation is fetched out using the Quantile-on-Quantile (QQ) tool.

### 5.1 Quantile cointegration test

Conventional cointegration tests use fixed cointegrating vectors, which might illustrate why cointegration across variables is never detected [24]. This investigation utilizes a quantile cointegration test introduced by Xiao [49] to eliminate biases in estimation. This test integrates time variations with the effect of diverse quantiles of the independent variable over the dependent variable to analyze long-run associations in a provisional data distribution. Because conventional cointegration tests have endogeneity problems, Xiao [49] reviewed them to fulfil the proposals of Saikkonen [50] by connecting dissolved cointegration residuals into lead-lag components [51].

In Equation (1), if α (τ) is considered a persistent vector, then the precise form of the cointegration regression might be stated as follows:

(1) $$X_{i}=\alpha +\alpha^{\prime }Y_{i}+\sum_{k=-s}^{k}\Delta Y_{i-k}^{\prime }\Pi_{k}+v_{i}$$

and

(2) $$Q_{\tau }^{X}\left(X_{i}{M_{i}}^{X},{M_{i}}^{y}\right)=\beta \left(\tau \right)+\alpha {\left(\tau \right)}^{\prime }Y_{i}+\sum_{k=-s}^{s}\Delta Y_{i-k}^{\prime }\Pi_{j}+F_{v}^{-1}\left(\tau \right)$$

In Equation (2), β(τ) denotes a drift component while α(τ) represents persistent parameters. $F_{v}^{-1}\left(\tau \right)$ represents the errors for different conditional data distribution quantiles. When the quadratic factor of the independent variable is considered, the cointegration regression is shown in Equation (3) as follows:

(3) $$Q_{\tau }^{X}\left(X_{i}{M_{i}}^{X},{M_{i}}^{y}\right)=\beta \left(\tau \right)+\alpha {\left(\tau \right)}^{\prime }Y_{i}+\delta {\left(\tau \right)}^{\prime }{Y_{i}}^{2}+\sum_{k=-s}^{s}\Delta Y_{i-k}^{\prime }\Pi_{k}+\sum_{k=-s}^{s}\Delta Y_{i-k}^{2}\Pi_{k}+F_{v}^{-1}\left(\tau \right)$$

To ascertain the cointegrating coefficients for the quantile cointegration test, ${\hat{V}}_{n}\left(\tau \right)=\left[\hat{\alpha }\left(\tau \right)-\hat{\alpha }\right]$ embodies in this investigation the null hypothesis (supremum rule). In this study, $Sup_{\tau }\left|V_{n}^{\prime }\left(\tau \right)\right|$ is used as a value of test statistics across complete quantile configurations. The test stat's vital values are determined by 1000 Monte Carlo simulations.

### 5.2 Quantile-on-quantile (QQ) technique

For our work, the QQ tool is applied as the superlative tool for constituting an association between our variables (*EP* and *CO*_*2*_) due to their asymmetrical distribution. OLS^3^ is resilient in situations not usually satisfied by intricate data. The OLS estimation can be biased because it coordinates a conditional average coefficient to consider multimodal data distribution. In the same way, the typical quantile regression (QR) process merely explores the explanatory variable's provisional average influences on the dependent variable's various quantiles [27]. Sim & Zhou [52] proposed the QQ technique as an extension of the prevailing QR model to handle many deficiencies in the traditional QR approach.

QQ is an excellent substitute for evaluating different quantiles of the independent and dependent variables, which integrates conventional QR and non-parametric estimations [52]. By examining the effect of the *EP* quantiles on the *CO*_*2*_ quantiles, this technique effectively resolves the issue of interdependence. Consequently, in our work, applying the QQ approach allows for identifying issues pertaining to the *EP-EQ* bond that may prove challenging to assess using conventional procedures like traditional ordinary least squares (OLS) or quantile regression (QR).

The fundamental model of our study in the form of non-parametric quantile regression, following by the studies of Zhao et al. [1] and Hassan et al. [19] can be expressed in Equation (4) as follows.

(4) $$C{O_{2}}_{t}=\alpha^{\varphi }\left(EP_{t}\right)+{\mu_{t}}^{\varphi }$$

*CO*_*2*_t and *EP*_t_ represent *CO*_*2*_ emission and energy poverty along time t, respectively. ɸ indicates the ɸ^th^ quantile for *CO*_*2*_. As we have no earlier awareness of the *EP-CO*_*2*_ nexus, the factor load α^ɸ^(.) can be considered anonymous. ${\mu_{t}}^{\theta }$ illustrates quantile error term alongside the ɸ^th^ quantile.

According to the idea of Cleveland [53], we estimate Equation (5) adopting local linear regression in the locality of *EP* asunder:

(5) $$\alpha^{\varphi }\left(EP_{t}\right)\approx \alpha^{\varphi }\left(EP^{\tau }\right)+\alpha^{\varphi^{\prime }}\left(EP^{\tau }\right)\left(EP_{t}-EP^{\tau }\right)$$

Here, α^ɸʹ^ exhibits the derivative of α^ɸ^ (*EP*_t_) in terms of *EP*_t_, which is also called partial derivative. α^ɸ^(*EP*^τ^) and α^ɸʹ^(*EP*^τ^) represent the functions of ɸ and τ, individually. α^ɸʹ^(*EP*^τ^) is referred to α_1_(ɸ,τ), and α^ɸ^(*EP*^τ^) is shown by α_0_(ɸ,τ). Consequently, the revised version of equation (5) can be written in the form of Equation (6) as follows:

(6) $$\alpha^{\varphi }\left(EP_{t}\right)\approx \alpha_{0}\left(\varphi ,\tau \right)+\alpha_{1}\left(\varphi ,\tau \right)\left(EP_{t}-EP^{\tau }\right)$$

The following QQ model is derived by establishing Equation (6) into Equation (4):

(7) $$C{O_{2}}_{t}=\frac{\alpha_{0}\left(\varphi ,\tau \right)+\alpha_{1}\left(\varphi ,\tau \right)\;\left(EP_{t}-\;{\text{EP}}^{\tau }\right)\;}{\left(*\right)}+u_{t}^{\varphi }$$

The empirical form of the QQ model is shown in equation (7). (*) identifies the conditional *EP* quantile. Equation (7) depicts the bond between the ɸ^th^ *EP* quantile and the τ^th^ *CO*_*2*_ quantile. The interrelation across several quantiles of *EP* and CO_2_ is characterized by parameters α_0_ and α_1_ and might fluctuate on the base of the quantiles of *EP* and *CO*_*2*_. The validation of the fundamental dependence structure between *EP* and *CO*_*2*_ is confirmed through Equation (7), which combines their respective distributions.

Despite the lack of additional control variables in the model, QQ surpasses other commonly used time-series data tools by effectively capturing the asymmetric linkage between *EP* and *CO*_*2*_ at multiple quantiles. This feature enhances the authenticity and reliability of the results compared to other conventional methods [54]. The selection of bandwidth (h) is vital in the optimization as it helps to elucidate the link between *EP* and *CO*_*2*_ quantiles. We embrace the minimization problem formed by Chu & Marron [55] as follows.

(8) $$Mi{n_{\delta_{0}}}_{\delta_{1}}\sum_{t=1}^{n}\rho_{\varphi }\left[C{O_{2}}_{t}-\delta_{0}-\delta_{1}\left(EP_{t}-EP^{\tau }\right)\right]L\left[\frac{M_{n}\left(EP_{t}\right)-\tau }{h}\right]$$

A shown in Equation (8), the quantile regression loss function is represented by $\rho_{\varphi }$. L (.) represents the Gaussian function that works as a weight parameter for the validity of the estimations by apportioning numerous weights to the data in neighbourhood of *EP*. The parameter ‘I’ represents the conventional indicator function, whereas h illustrates the bandwidth parameter.

In Kernel regression, the bandwidth functions as a smoothing parameter by limiting bias and variation. Higher bandwidth value causes skewed estimations, while a smaller bandwidth leads to higher variance [52]. Thereby, achieving the proper balance between bias and variance is critical. Thereby, it is essential to establish stability between variance and bias. Following Shahzad et al. [51], we adopt a bandwidth limit of h = 0.05 (5%).

### 5.3 Robustness of the QQ technique

The QQ model could produce the conventional QR estimation by approving correct considerations for several quantiles of the explanatory variable (*EP*). Regardless of the certainty that its coefficients are only indexed by ɸ, the QR approach could portend the effect of ɸ^th^ *EP* quantile on *CO*_*2*_ in this research. Contrary to the QR methodology, the QQ regression calculates the impact of the ɸ^th^ *EP* quantile on the τ^th^ *CO*_*2*_ quantile, indexing the quantile components using both ɸ and τ, thereby generating more classified data. Thus, the QR coefficients could be estimated by attaining the mean of the coefficients of the QQ model alongside τ. The slope coefficient of the QR regression is examined by $\gamma_{1}\left(\theta \right)$, and it is used to estimate the effect of *EP* on multiple *CO*_*2*_ quantiles as described in the following:

(9) $$\gamma_{1}\left(\varphi \right)\equiv {\bar{\hat{\alpha }}}_{1}=\frac{1}{s}\sum_{\tau }{\hat{\alpha }}_{1}\left(\varphi ,\tau \right)$$

In Equation (9), s = 19 illustrates the number of quantiles, and τ denotes the quantile range, which spans from 0.05 to 0.95. We might test the robustness of the QQ methodology by correlating the estimated QR coefficients to the τ-averaged QQ coefficients.

## 6 Findings and discussion

The current section explains the investigation's preliminary and main outcomes along with a thorough discussion.

### 6.1 Initial outcomes

Table 3 displays the descriptive statistics of *EP* and *CO*_*2*_ for the selected countries in our study.

**Table 3:** Descriptive statistics values for *EP* and *CO*_*2*_.

Economies	Mean	Min.	Max.	Std. Dev.	J-B Stats	ADF(Level)	ADFΔ
Panel 1: Energy Poverty (*EP*)^4^							
India	28.76	4.30	46.99	12.79	3.30*	−0.91	−6.18*
Pakistan	29.31	27.21	30.67	0.67	4.74*	−1.92	−5.68*
Bangladesh	48.90	8.19	78.85	19.85	6.59*	−1.40	−4.24*
Nepal	45.92	6.08	82.10	25.32	3.90*	−1.36	−5.61*
Maldives	7.37	0.09	20.10	7.14	2.20*	−2.15*	−3.51**
Afghanistan	60.31	2.30	98.88	34.41	4.20*	−1.70	−6.14*
Sri Lanka	18.28	0.43	36.40	10.86	4.60*	−1.55	−5.66*
Bhutan	35.90	0.02	73.06	25.99	3.14*	−1.32	−4.31*
**Panel 2: Carbon Dioxide Emissions (*CO***_***2***_**)**							
India	1457178	776720	2434520	545754	2.57*	−1.72	−5.62*
Pakistan	132677	85820	208370	34217.34	3.07*	−5.34*	−6.28*
Bangladesh	43320.43	16820	82760	20965.20	4.06*	−1.96	−3.93*
Nepal	4703.91	1960	12030	2845.75	5.51*	−1.87	−4.12*
Maldives	906.08	280	1910	479.15	3.18*	−2.08*	−5.72*
Afghanistan	4501.73	770	12260	3738.53	2.40*	−1.94	−3.72**
Sri Lanka	14041.65	8340	23310	4382.65	2.38*	−1.91	−3.73**
Bhutan	596.95	280	1380	348.30	1.47	−1.68	−4.46*

Note:* and ** display the significance levels at 1% and 5%, individually.

Bhutan is at the top of the list due to reaching its minimum level of *EP*, which shows that only 0.02% of the population has no electricity access. The maximum *EP* level during the study period reached 73.06%. Maldives is placed second, with the minimum level of *EP* (0.09%), reaching its maximum level of 20.10. Sri Lanka and Afghanistan are ranked third and fourth, having a minimum *EP* level of 0.43 and 2.30, respectively. If we see the *EQ*, India is the most polluted country with an average *CO*_*2*_ level of (1457178) kiloton (kt) spanning from 776720 to 2434520. Pakistan holds the second rank, with an average *CO*_*2*_ of (132677) kt spanning from 85820 to 208370. Bangladesh and Sri Lanka are rated third and fourth, having mean *CO*_*2*_ values of 43320.43 to 14041.65 kt.

The results of Jarque-Bera (J-B) test indicate that the dataset, consisting of *EP* and *CO*_*2*_, follows a non-normal distribution across most of the studied economies. An exception to this trend is observed in Bhutan, where *CO*_*2*_ exhibit a normal distribution. This prevalence of non-normal distribution in our dataset reinforces the appropriateness of employing the QQ method in our analysis, as Shahbaz et al. [54]. Additionally, the ADF^5^ test reveals that most variables achieve stationarity after the first difference. Consequently, we have adapted our data series to this stationary state by converting our variables into their first differences, in line with the methodologies utilized by Shahbaz et al. [54] and Shahzad et al. [51].

According to Table 4, *EP* and *CO*_*2*_ are significantly and positively connected with each other according to the correlation coefficients for all nations. Pakistan specifies the biggest value of correlation (0.84), chased by Sri Lanka (0.83), Bangladesh (0.80), and Nepal (0.75).

**Table 4:** Correlation between *EP* and *CO*_*2*_.

Economy	Correlation	t-Stats	p.value
India	0.67	8.60*	0.000
Pakistan	0.84	10.60*	0.000
Bangladesh	0.80	4.90*	0.000
Nepal	0.75	9.34*	0.000
Maldives	0.68	8.92*	0.000
Afghanistan	0.74	4.07*	0.000
Sri Lanka	0.83	20.30*	0.000
Bhutan	0.65	10.32*	0.000

Note:’*’ expresses the significance level at 1%.

### 6.2 Key findings

The outcomes of the quantile cointegration test are given in Table 5 τ referring to the τ^th^ quantile of *EP*. The coefficients of the supremum norm (α and γ) are acquired from equation (3), indicating parameter consistency.

**Table 5:** Findings of quantile cointegration test (*EP* and *CO*_*2*_).

Economies	Coefficients	Sup_τ_ |V_n_(τ)|	C1	C5	C10
India *EP* vs. *CO*_*2*_	α	6237.60	5683.95	4686.52	3781.77
	γ	3271.95	2693.70	2181.72	1849.40
Pakistan *EP* vs. *CO*_*2*_	α	8315.20	5283.22	3137.01	2521.36
	γ	178.62	110.40	54.86	38.33
Bangladesh *EP* vs. *CO*_*2*_	α	68591.32	58356.33	57302.20	54881.73
	γ	2452.63	1493.20	1445.40	1431.10
Nepal *EP* vs. *CO*_*2*_	α	3930.92	3769.26	248.52	205.97
	γ	166.71	156.80	48.09	44.78
Maldives *EP* vs. *CO*_*2*_	α	539.42	324.35	290.75	236.57
	γ	288.97	196.90	128.70	97.38
Afghanistan *EP* vs. *CO*_*2*_	α	1837.70	1546.78	1041.70	991.86
	γ	952.77	689.60	496.70	345.80
Sri Lanka *EP* vs. *CO*_*2*_	α	1244.70	934.78	549.07	207.72
	γ	786.80	586.95	496.95	373.70
Bhutan *EP* vs. *CO*_*2*_	α	7115.30	3491.11	3081.10	2224.39
	γ	608.44	302.88	212.20	116.10

**Note:** A grid consisting of 19 equally spaced quantiles spanning from 0.05 to 0.95 is utilized to compute t-statistics. Additionally, the maximum norm values for the parameters γ and α, together with their critical boundaries at the significance levels of 1% (C1), 5% (C5), and 10% (C10), are displayed.

The findings obtained from the quantile cointegration test display variations in the long-run relationship between *EP* and *CO*_*2*_ among different quantiles within each economy. The coefficients (α and γ) exhibit higher supremum norm scores compared to the corresponding critical bounds (C1, C5, and C10), which verifies an asymmetric long-run linkage between the variables in all economies.

Fig. 1 depicts the slope measures α_1_ (ɸ, ***τ***), which disclose the impact of ɸ^th^ *EP* quantile on ***τ***^th^ *CO*_*2*_ quantile using diverse values of ɸ and ***τ*** in the South Asian countries. **India** in Fig. 1(a) and Afghanistan in Fig. 1(f), the positive and powerful effect of *EP* on carbon dioxide is leading. A positive powerful *EP-CO*_*2*_ bond is exhibited in the divisions that incorporate complete *EP* quantiles with the mid-lower to topmost *CO*_*2*_ quantiles. The notably robust and positive bond submits that the *EP* deteriorates the environment by maximizing *CO*_*2*_ at rising pollution ranks. However, a powerful negative *EP-CO*_*2*_ tie is also discovered in the locations, which meld overall *EP* quantiles with low to moderately low quantiles of *CO*_*2*_ (0.05–0.30). The positive *EP-CO*_*2*_ nexus in Afghanistan and India is supported by Bilgili et al. [22], who claim that *EP* degrades *EQ* in Asian countries. This strong inverse linkage proposed that the *EP* boosts the *EQ* by declining *CO*_*2*_ at low ranks of *CO*_*2*_. Though, a fragile positive linkage between *EP* and *CO*_*2*_ is also discovered in India, where *EP* quantiles correlate with mid-low quantiles of emissions (0.30–0.35).

**Fig. 1:** **Quantile-on-Quantile (QQ) estimations of the slope coefficient** α_1_ (ɸ, ***τ***) Note: The z-axis displays the slope coefficients α_1_(ɸ, ***τ***), while the x-axis represents the EP quantiles and the y-axis represents the *CO*_*2*_ quantiles. The colors depicted on the graphs' right side points out the slope coefficients, ranging from blue (reflecting lower values) to red (pointing upper values). A rich red shade signifies a strong positive *EP-CO*_*2*_ connection, whereas a dark blue tone suggests a strong inverse relationship. Likewise, a mild red color indicates a weak positive linkage, whereas a fainter blue hue asserts an inverse and weak *EP-CO*_*2*_ association. This visible representation is indicative of evaluating the intensity and orientation of the *EP-CO*_*2*_ connection across multiple contexts. (For interpretation of the references to color in this figure legend, the reader is referred to the Web version of this article.)

In Fig. 1(b), **Pakistan,** shows a positive powerful *EP-CO*_*2*_ nexus is developed throughout the vicinities, which incorporate complete *EP* quantiles with the bottommost to median-high quantiles of carbon emissions (0.05–0.70). This particular positive significant junction states that the *EP* deteriorates the *EQ* by maximizing carbon dioxide at rising pollution ranks. Moreover, a positive and insignificant/weak bond between *EP* and *CO*_*2*_ is also developed in the portions, which correlate overall quantiles with mid-high to topmost *CO*_*2*_ quantiles (0.75–0.95). Though, the negative powerful *EP-CO*_*2*_ attachment is also prevailed across the chunks, which tie top *EP* quantiles and lowest *CO*_*2*_ quantiles. This powerful inverse interconnection proposed that the *EP* boosts the *EQ* by lessening *CO*_*2*_ at the top ranks of *EP* and low levels of pollution. In Fig. 1 (c), **Bangladesh** shows a positive impact of *EP* on *CO*_*2*_. A positive vigorous *EP-CO*_*2*_ interdependence is discovered between the zones, which amalgamate all *EP* quantiles with the bottom to moderate emissions quantiles (0.05–0.50). This notably robust and positive conjunction demonstrates that *EP* degrades the *EQ* by maximizing *CO*_*2*_ at uplift pollution grades. Moreover, a feeble and positive *EP-CO*_*2*_ conjunction is discovered in the chunks incorporating whole *EP* quantiles with medium to upmost quantiles of pollution (0.55–0.95). It indicates that *EP* is insignificantly correlated with *CO*_*2*_ at rising pollution grades. The outcomes are consistent with Kousar & Shabbir [46], who found a positive impact of *EP* on *CO*_*2*_ in Pakistan.

In Fig. 1(g), **Sri Lanka** shows a a positive and vigorous effect of *EP* on *CO*_*2*_. This positive and robust relationship between *EP* and carbon emissions is consistently identified across various locations, encompassing all quantiles of *EP* combined with both lower to mid-high and upper quantiles of *CO*_*2*_. This mainly powerful positive linkage suggests that *EP* significantly lowers the *EQ* by maximizing carbon dioxide at bottommost to moderate and upmost pollution ranks. In the regions where high *EP* quantiles overlap with mid-range carbon quantiles (0.65–0.80), a weak negative correlation between *EP* and *CO*_*2*_ emerges. In Fig. 1(h), **Bhutan** exhibits a prominent and positive nexus between *EP* and *CO*_*2*_, where a positive and powerful correlation between *EP* and *CO*_*2*_ is found in chunks that unify entire quantiles of *EP* with the median to higher *CO*_*2*_ quantiles (0.50–0.95). This robust positive association signifies that *EP* negatively impacts *EQ* by diminishing *CO*_*2*_ as pollution levels increase. A moderate positive link across *EP* and *CO*_*2*_ is also matured across the districts that unify all *EP* quantiles with extremely low to median carbon emissions (0.05–0.45). The domination of the positive and powerful effect of *EP* on *CO*_*2*_ is supported by Bilgili et al. [22], who establish that *EP* degrades *EQ* in Asian nations.

In Fig. 1(d), there exists a mixed bond between *EP* and *CO*_*2*_ in **Nepal.** A positive, vigorous *EP-CO*_*2*_ linkage is discovered between the spots that tie the lowest to moderate *EP* quantiles (0.05–0.50) and full *CO*_*2*_ quantiles. This mainly powerful and positive relation proposes that the *EP* boosts *CO*_*2*_ at times of lower to median ranks of *EP*. Furthermore, a fragile positive *EP-CO*_*2*_ nexus is discovered in the localities that tie moderately high *EP* quantiles (0.75–0.85) with complete quantiles of carbon emissions. Though, an inverse and powerful *EP-CO*_*2*_ bond is also discovered in the zones, which combine moderately high and highest *EP* quantiles (0.55–0.70 & 0.90–0.95) with complete quantiles of *CO*_*2*_. Like Nepal, the **Maldives** exhibits a mixed alliance between *EP* and *CO*_*2*_ (as shown in Fig. 1(e)). Among various locations, a positive and strong connection is identified between *EP* and *CO*_*2*_, particularly when combining all *EP* quantiles with medium to highest *CO*_*2*_ quantiles (0.55–0.95). This particularly powerful positive relation proposes that the *EP* raises *CO*_*2*_ in the Maldives at moderate to high levels of *CO*_*2*_. It entails that *EP* lowers *EQ* by augmenting *CO*_*2*_ in times of higher pollution ranks. Though, a powerful negative *EP-CO*_*2*_ linkage is discovered in the vicinities linking total *EP* quantiles with small to moderate *CO*_*2*_ quantiles. It exhibits that *EP* boosts *EQ* by decreasing the grades of *CO*_*2*_ at the time of lower to medium grades of *CO*_*2*_. The findings of the mixed relationship between *EP* and *CO*_*2*_ are supported by the study of Filippidis et al. [43], who revealed a time-varying junction between *EP* and *CO*_*2*_ by discovering an inverted U-shaped Environmental Kuznets curve. Filippidis et al. [43] also claim that the influence of *EP* can vary depending on economic circumstances. Moreover, this mixed correlation could be attributable to distinctive features like energy consumption, energy efficiency, population growth patterns, and technical expansions in these countries.

Drawing from the analysis presented in Fig. 1, Table 6 delves into the correlation between *EP* and *CO*_*2*_ across a range of chosen economies. It uncovers a pronounced positive correlation in six out of eight of these economies, highlighting a significant link where changes in *EP* levels are closely mirrored by increased *CO*_*2*_. This trend underscores the direct effect of *EP* on environmental factors. However, this relationship is not universally applicable, as evidenced in the cases of Nepal and the Maldives. In these countries, the data indicates a more intricate and varied correlation between *EP* and *CO*_*2*_. This mixed pattern suggests that local factors, possibly including specific environmental policies and economic circumstances, perform a crucial part in building the unique interplay between energy usage and its environmental repercussions in several regions.

**Table 6:** Summary of Findings (Relationship b/w Numerous Quantiles of *EP* and *CO*_*2*_).

Nations	*EP* Quantiles	*CO*_*2*_ Quantiles of	Relationship b/w quantiles	Dominant connection
India	Overall quantiles	Lower-middle to highest quantiles	Powerful positive	Powerful positive
	Whole quantiles	Lower to low-mid quantiles	Strong inverse	
	All quantiles	Lower-mid quantiles	Weak positive	
Pakistan	Whole quantiles	Low to mid-high quantiles	Powerful positive	Powerful positive
	Overall quantiles	High-mid to top quantiles	Feeble positive	
	Top quantiles	Lowest quantiles	Inverse powerful	
Bangladesh	Total quantiles	Bottom to medium quantiles	Positive powerful	Powerful positive
	Total quantiles	Mid to topmost quantiles	Weak positive	
Nepal	Bottom to mid quantiles	Full quantiles	Powerful positive	Mixed correlation
	Upper-mid quantiles	Total quantiles	Feeble positive	
	Upper-middle and highest quantiles	Entire quantiles	Powerful inverse	
Maldives	Complete quantiles	Medium to top quantile**ѕ**	Powerful positive	Mixed correlation
	Whole quantile**ѕ**	Low to middle quantiles	Powerful negative	
Afghanistan	Complete quantile**ѕ**	Low-mid to highest quantile**ѕ**	Positive powerful	Powerful positive
	Entire quantile**ѕ**	Low to low-mid quantiles	Strong inverse	
Sri Lanka	Entire quantiles	Bottom to high-middle and top quantiles	Strong positive	Positive powerful
	Total quantiles	Higher-middle quantile**ѕ**	Strong inverse	
Bhutan	Complete quantiles	Middle to higher quantiles	Strong positive	Powerful positive
	Complete quantiles	Bottom to medium quantiles	Moderate positive	

### 6.3 Robustness of the QQ methodology

By comparing the QQ estimations with the QR calculates, we can determine their level of similarity. Fig. 2 serves as confirmation for the prior conclusions of the QQ technique. The graphs demonstrate that the slope parameters’ mean QQ assessments align with the pattern observed in the QR estimations for all selected economies.

**Fig. 2:** Validating the Robustness of the QQ Tool by Relating QQ and QR Tool Note: The estimations for the parameters of traditional QR regression and the averaged-QQ parameters plotted against different *CO*_*2*_ quantiles.

Fig. 2 reveals that Pakistan in Fig. 2(b), India in Fig. 2(a), Bangladesh in Fig. 2(c), Nepal in Fig. 2(d), Maldives in Fig. 2(e), Afghanistan in Fig. 2(f), Bhutan in Fig. 2(h), and Sri Lanka in Fig. 2(g) have a positive link between *EP* and *CO*_*2*_. Moreover, Nepal in Fig. 2(d) and Maldives in Fig. 2(e) have mixed outcomes by demonstrating a mixture of both negative and positive correlations within numerous *EP-CO*_*2*_ quantiles. Additionally, in this analysis show that *EP* and *CO*_*2*_ vary in entire selected countries. The coefficients’ extents elucidate that the effect of *EP* on *CO*_*2*_ is substantially greater in Sri Lanka, Nepal, and Pakistan. Moreover, in Bangladesh and Maldives, the efficacy of *EP* is absolutely down.

### 6.4 Discussion of results

Generally, the consequences suggest a positive *EP-CO*_*2*_ association in majority of our selected nations. By supporting the hypothesis, *EP* has been identified to be a cause of growing pollution in 6 out of 8 chosen economies, by confirming the hypothesis, as do other studies, such as Bilgili et al. [22], Okushima [18], and Hassan et al. [19] that propose that *EP* lowers *EQ* by enhancing *CO*_*2*_. The positive *EP-CO*_*2*_ relation in our findings is also consistent with those of Ehsanullah et al. [20] for G7 economies, Qin et al. (2021) for E−7 nations, Hassan et al. [19] for and Zhao et al. (2021) for China.

Within varied the data distribution quantiles, the bond between *EP* and *CO*_*2*_ varies considerably in the nations we analyzed. This conduct is maintained by the empirical research of Akram et al. [56], who identified a time-varying asymmetric energy efficiency-*CO*_*2*_ interconnection. Furthermore, Nepal and Maldives have mixed outcomes throughout numerous *EP-CO*_*2*_ quantiles. The mixed *EP-CO*_*2*_ affiliation in these nations is persistent with Filippidis et al. [43], who disclosed a time-varying *EP-CO*_*2*_ association by discovering an inverted U-shaped Environmental Kuznets curve. As countries initially develop, their *CO*_*2*_ tends to increase, but beyond a certain level of economic development, they start to decrease. Therefore, it is reasonable to expect mixed outcomes in Nepal and Maldives as they fall at different points along this curve. Filippidis et al. [43] also claim that the influence of *EP* can vary depending on economic circumstances. Economies with different economic conditions may have varying levels of reach to cleaner energy sources and technologies, which can affect their carbon emissions. Nepal and Maldives, despite having different economic circumstances, both face challenges related to *EP* and have different levels of access to energy resources. These differences can contribute to the mixed outcomes observed. Moreover, several factors can contribute to the diverse correlation between *EP* and *CO*_*2*_ in these nations. Energy consumption patterns play a crucial part in determining *CO*_*2*_. The type and amount of energy sources used, namely fossil fuels or renewable energy, can significantly impact a country's carbon footprint. Differences in energy efficiency practices also influence *CO*_*2*_. Countries with more efficient energy usage tend to have lower emissions. Population growth trends can also affect the correlation between *EP* and *CO*_*2*_. Rapidly growing populations may pressure on energy resources and infrastructure, potentially producing higher *CO*_*2*_. On the other hand, technological advancements can enable more sustainable and cleaner energy solutions, reducing carbon emissions even in the presence of *EP*.

As discussed before, the impact of *EP* fluctuates extensively between quantiles and throughout the sample. By way of illustration, the highest quantiles of *CO*_*2*_ have an extra powerful connection with *EP* (in India, Maldives, Afghanistan, Sri Lanka, and Bhutan). It means that at high *CO*_*2*_ levels, *EP* significantly accelerates the level of *CO*_*2*_. In other words, as *CO*_*2*_ levels increase to higher quantiles, the influence of *EP* on *CO*_*2*_ becomes more pronounced. The results are also backed by Filippidis et al. [44], who suggest the level of *EP* is beneficial to *EQ* just up to a specific threshold, after which more *EP* is harmful to the ecosystem. This suggests that there is an optimal level of *EP* that benefits the ecosystem, but exceeding this threshold leads to negative consequences. Therefore, the claim that the highest quantiles of *CO*_*2*_ exhibit a stronger connection with *EP*, leading to an acceleration of *CO*_*2*_ levels, is plausible and in line with the understanding that excessive pollution can have detrimental effects on the environment.

The *EP-CO*_*2*_ slope coefficients fluctuate throughout nations, confirming that the *EP-CO*_*2*_ correlation is linked to the compass and symbol of macroeconomic shocks and the certain economic period (recession or boom) that determines *CO*_*2*_. Economic activity tends to contract during a recession, guiding to lessened industrial production and low consumption of energy. This could result in a decrease in *CO*_*2*_ and subsequently weaken the relationship between *EP* and *CO*_*2*_. On the other hand, during a boom period, economic activity expands, leading to increased industrial production and higher energy consumption. This may contribute to higher *CO*_*2*_ and strengthen the relationship between *EP* and *CO*_*2*_. Furthermore, different nations may have varying levels of environmental regulations, technological capabilities, and energy sources. These factors can influence the extent to which *EP* affects *CO*_*2*_. Countries with less stringent regulations or reliance on fossil fuels may experience a stronger connection between *EP* and *CO*_*2*_, in contrast countries with stricter regulations or greater adoption of renewable energy sources may exhibit a weaker relationship. Consequently, our sample nations encounter rare conditions that panel data methodologies cannot analyze. Therefore, we have studied every economy distinctly and profoundly in rank to absolutely hold its exclusive qualities.

## 7 Conclusion and policy implications

This paper has evaluated the nonlinear *EP-EQ* nexus in South Asian economies using data from 1996 to 2019. We have applied the QQ tool that independently evaluates time-series dependence in every economy to offer international yet nation-specific details concerning the *EP-CO*_*2*_ nexus. According to the estimation, *EP* degrades *EQ* in most of selected economies at specific data distribution quantiles.

The implications of our findings have wide-ranging effects on South Asian countries, offering policymakers new viewpoints on the bond between energy production and environmental quality. Policymakers should exercise care when interpreting the results of this study. Compared to other areas, the progress in access to electricity in South Asian nations over the last 20 years has been significant, and millions of people in these nations now have access to electricity. There has been a dramatic reduction in *EP* in terms of access to electricity. Although growing urbanization increases electrification in this region, government actions also aid the process. As of 2021, the remaining population that suffers from *EP* in conditions of reach to electricity is found in rural areas of South Asia. Governments of South Asian countries should play a critical role in sparking national policy actions and international collaboration to relieve *EP* in terms of access to power. Different financial approaches to assist poor households are significantly enhance the electrification rate. Grid-based electricity derived from renewable energies, specifically hydropower, should be prioritized to reduce *EP* and *CO*_*2*_ in South Asia. Stand-alone small house systems based on indigenous renewable energies (i.e., solar PV and wind) should meet the demands of the un-electrified areas in these countries for the very remote places where connecting to the grid is either unfeasible or uneconomical.

The key observation from the global energy system of production and consumption is that most energy is intended for industrial use rather than private consumption. Private residents utilize around a quarter of the total energy supply. Energy access is geared toward private citizens rather than industry. It advocates for the global energy system to prioritize humans above multinational corporations. We must give access to cheap, sustainable, and clean energy for all, according to the definition of SDG-7, with the UN placing four specific demands on energy access (reliable, affordable, sustainable, and contemporary). Energy access is a poverty-driven issue for policymakers. It is about providing electricity and heating to the most vulnerable members of our global society. Decision-makers must assess how their current and future energy investments will enable or hinder solutions. Securing resources for net consumers, suppliers, and those without access still needs to be improved for providing sustainable energy and, eventually, a more balanced system. We must also examine the long-term consequences of our energy decisions. If sustainable energy offers zero or low-carbon solutions, a fair global energy system requires rebalancing all three characteristics: accessibility, availability, and sustainability. Energy efficiency improvement in houses can have various unexpected effects, including low indoor air quality, an increased risk of midsummer overheating, and building moisture hazards.

Most of our selected countries are abundant in renewable energy sources like hydropower, solar, and wind. Incentives and assistance for renewable/clean energy generation and technology are crucial for increasing energy access and improving *EQ*. Technological advancement directs production through resource efficiency and improves *EQ* by contributing to *CO*_*2*_ reduction. Renewable sources create clean energy that is important for human well-being while also assisting in solving the problem of limited electricity access in distant locations of underdeveloped economies. Furthermore, governments should provide subsidies to replace wood fuel with biogas. International organizations and policy authorities should provide more funds, loans, and subsidies for renewable energy. Building capacity is required to minimize the cost of new installations and electricity consumption to make energy more affordable to the general population. Energy planners must consider restricted financial restrictions and the long-term prospects that clean energy provides for individuals residing in rural regions. Most countries in the modern period rely on fossil fuels and hydropower. As a result, provincial and federal governments must diversify their energy sources (solar, wind, biomass, and geothermal). These methods will enhance electricity output, leading to lower electricity costs. The donor countries and international community must assist our selected countries in building their eco-friendly energy policies. Donor countries must promote the transfer of innovative technologies and collaborate with beneficiary economies on international energy finance programs.

Our research has identified some restraints that can supervise forthcoming investigations on ongoing topic. The conclusions obtained by this study are relevant to many of our chosen countries, together with other economies that are tackling environmental issues. This work emphasizes a particular set of economies (South Asia). However, varying groups of economies or vicinities could affect the estimations differently. Forthcoming studies would help improve our comprehension of the *EP-EQ* link against the background of the European, Middle East, Sub-Saharan African, and Latin American economies. For upcoming studies, an analysis that encompasses fieldwork, household conversations, and extensive data (if practical) to consider the advancement of *EP* reduction would give crucial details in identifying the expertise of *EP* and contribute to government policy measures, trends, and initiatives to expand *EQ*. In our research, we looked at the effect of *EP* on *CO*_*2*_. More research is vital to conclude the effect of *EP* on other components of GHG emissions (SO_2_, N_2_O, and CH_4_) and the ecological footprint.

## Human and animal rights

No human or animals were harmed to do this research.

## Availability of data

The datasets used during the current study are available from the corresponding author on reasonable request.

## Funding

No funding was received for conducting this study.

## Ethics approval and consent to participate

N/A.

## Consent for publication

N/A.

## CRediT authorship contribution statement

**Jifa Rao:** Writing – original draft, Formal analysis, Conceptualization. **Sajid Ali:** Writing – review & editing, Writing – original draft. **Raima Nazar:** Writing – original draft, Methodology. **Muhammad Khalid Anser:** Writing – original draft, Software.

## Declaration of competing interest

The authors declare that they have no known competing financial interests or personal relationships that could have appeared to influence the work reported in this paper.

## Footnotes

4 *EP* is measured by calculating the population without access to electricity (%).

## Footnotes

1 India, Pakistan, Bangladesh, Nepal, Maldives, Afghanistan, Sri Lanka, and Bhutan.

2 India, Pakistan, Bangladesh, Nepal, Maldives, Afghanistan, Sri Lanka, and Bhutan.

3 Ordinary Least Squares.
